# *De novo* transcriptome analysis and identification of reproduction control genes from the red palm weevil *Rhynchophorus ferrugineus*

**DOI:** 10.1371/journal.pone.0251278

**Published:** 2021-05-24

**Authors:** Khawaja Ghulam Rasool, Khalid Mehmood, Mureed Husain, Muhammad Tufail, Waleed Saleh Alwaneen, Abdulrahman Saad Aldawood

**Affiliations:** 1 Economic Entomology Research Unit, Plant Protection Department, College of Food and Agriculture Sciences, King Saud University, Riyadh, Saudi Arabia; 2 Institute of Plant Protection, Faculty of Agriculture and Environmental Sciences, MNS-University of Agriculture, Multan, Pakistan; 3 Ghazi University, Dera Ghazi Khan, Punjab, Pakistan; 4 National Center for Agricultural Technology (NCAT), King Abdulaziz City for Science and Technology (KACST), Riyadh, Saudi Arabia; Harran Üniversitesi: Harran Universitesi, TURKEY

## Abstract

Recent attacks by the red palm weevil, *Rhynchophorus ferrugineus* (Olivier), have become a severe problem for palm species. In present work, fat body transcriptome of adult female red palm weevil was analyzed, focusing on the identification of reproduction control genes. Transcriptome study was completed by means of next-generation sequencing (NGS) using Illumina Hiseq 2000 sequencing system. A total of 105,938,182 raw reads, 102,645,544 clean reads, and 9,238,098,960 clean nucleotides with a guanine–cytosine content of 40.31%, were produced. The processed transcriptome data resulted in 43,789 unique transcripts (with mean lengths of 1,172 bp). It was found that 20% of total unique transcripts shared up to 80%–100% sequence identity with homologous species, mainly the mountain pine beetle *Dendroctonus ponderosae* (59.9%) and red flour beetle *Tribolium castaneum* (26.9%). Nearly 25 annotated genes were predicted to be involved in red palm weevil reproduction, including five vitellogenin (Vg) transcripts. Among the five *Vg* gene transcripts, one was highly expressed compared with the other four (FPKM values of 1.963, 1.471, 1.028, and 1.017, respectively), and the five *Vg* gene transcripts were designated as *RfVg*, *RfVg-equivalent1*, *RfVg-equivalent2*, *RfVg-equivalent3*, and *RfVg-equivalent4*, respectively. The high expression level of *RfVg* verified by RT-polymerase chain reaction analysis suggested that *RfVg* is the primary functional *Vg* gene in red palm weevil. A high similarity of *RfVg* with other Coleopterans was also reflected in a phylogenetic tree, where *RfVg* was placed within the clade of the order Coleoptera. Awareness of the major genes that play critical roles in reproduction and proliferation of red palm weevil is valuable to understand their reproduction mechanism at a molecular level. In addition, for future molecular studies, the NGS dataset obtained will be useful and will promote the exploration of biotech-based control strategies against red palm weevil, a primary pest of palm trees.

## Introduction

The red palm weevil (RPW), *Rhynchophorus ferrugineus* (Olivier) (Coleoptera: Dryophthoridae) has strong invasion capability and within the last few decades have become invasive in more than 27 countries around the globe [1]. The RPW has become the most devastating pest of palm family, including economically valued palms, such as the date palm *Phoenix dactylifera*, coconut palm *Cocos nucifera*, and African oil palm *Elaeis guineensis* [2–4]. The female RPW can deposit 270–396 eggs throughout the lifespan [5]. The larvae feed and damage the host palm until a severe infestation occurs in the tree. RPW mostly feed on young palm trees, causing high economic losses [6]. The reproduction success of oviparous species, including insects, depends on reproduction control genes expression, particularly the genes involved in vitellogenin (Vg) biosynthesis and its uptake [7–9]. The Vgs are egg yolk protein precursors and play a vital role in the proliferation of oviparous organisms.

In recent decades, scientists have studied the basic ecology and biology of RPW [1, 10–12] and have examined various control strategies, including the use of chemicals, entomopathogens, and pheromone traps [13–15]. However, none of these strategies examined so far have been singly successful in controlling the spread of RPW. The reason for this is probably the concealed nature of pests reproducing inside palm trees. Unfortunately, the mechanisms behind the molecular regulation of reproduction of this species remain unclear. Therefore, awareness of the major genes that play a critical role in its reproduction and proliferation could be valuable by providing the rudimentary knowledge of the reproduction mechanisms of RPW at a molecular level.

The rapid progress and convergence of modern techniques from different areas of science have resulted in the enrichment of the fields of genetics and molecular sciences. Next-generation sequencing (NGS) is an efficient and economical technology used for identification of large numbers of expressed genes in a specific tissue, and confirms the biological, physiological, and molecular properties of the tissue. The use of NGS is very effective for discovering novel genes and determining gene structures and functions [16, 17]. This *de novo* transcriptome sequencing technology has been successfully demonstrated in several insects, including the migratory locust *Locusta migratoria* [18], oriental fruit fly *Bactrocera dorsalis* [19], noctuid moth *Spodoptera littoralis* [20], RPW *R*. *ferrugineus* [21], brown plant hopper *Nilaparvata lugens* [22], and almond moth *Ephestia cautella* [23].

Thus, to isolate RPW reproduction control genes, the transcriptome of female fat body tissue was sequenced and analyzed using an Illumina Hiseq 2000 NGS platform. Although transcriptome and genome resources are accessible from several Coleopteran insects [24–28], the transcriptome sequence of RPW fat body tissue will expand the genomic resources available to researchers worldwide. The transcriptome analysis in the current study resulted in 105,938,182 raw reads with a guanine–cytosine (GC) content of 40.31%. High-quality reads were assembled into 43,789 unique transcripts or unigenes. The results of functional annotation revealed 25 genes that were likely involved in RPW reproduction, including *Vg* and other important genes such as: apolipophorin III, low-density lipoprotein receptor, and the chorion protein. The analysis of the fat body transcriptome provides extensive information about the genes involved in biological, physiological, and metabolic processes of the RPW and may facilitate future molecular studies, especially of Coleopteran animals, and even promote development of control tactics against invasive species, particularly the RPW.

## Materials and methods

### Ethics statement

The red palm weevil adults were collected directly from the date palm orchard, Riyadh region, Saudi Arabia. We declare that red palm weevil was not collected from the public parks or protected areas. Moreover, it is not an endangered species.

### Rearing of the red palm weevil

RPW different stages (larva, pupa, and adult) were initially collected from infested date palm trees in Dirab, Kingdom of Saudi Arabia (24.4164°N, 46.5765°E). Adult RPW were kept in plastic boxes containing a piece of cotton saturated with 10% sugar solution [10]. The laid eggs were collected and transported on wet filter paper into small plastic cups. Larvae were provided artificial diet (250 g per 5 larvae) in a plastic box. Finally, the last instar larvae were moved for pupation into a piece of sugarcane. RPW colonies were maintained in the growth chamber at 25°C ± 1°C and 70% ± 5% relative humidity.

### Fat body tissue preparation

A total of 25 (1–5 days old) virgin adult females were selected from the colony for fat body tissue preparations. The insects were dissected using fine microscissors in phosphate-buffered saline (pH 8.0) [29]. The fat body tissues were isolated, froze immediately in liquid nitrogen, and stored at −80°C. Finally, the fat body samples were transferred to RNAlater (RNA Stabilization Solution, Ambion, USA) and sent to Beijing Genomics Institute, China, for transcriptome analysis.

### RNA isolation and cDNA synthesis

Total RNA was extracted from RPW fat body tissues (~800 mg) using Tri-RNA reagent (Favorgen Biotech CORP, Taiwan). The RNA integrity number 28S/18S ratio and sample size were determined using an Agilent 2100 Bioanalyzer and Agilent RNA 6000 Nano Kit and DNase treatment was done to elude genomic DNA contamination. Finally, the purity was assessed by using NanoDrop. The total volume of 80 μL RNA samples with a concentration of 488 ng/μL were used to synthesize cDNA. The Superscript II Reverse Transcription kit (Invitrogen) was used to generate first-strand complementary DNA from mRNA. To synthesize second-strand cDNA, second-strand master mix was added in the first-strand cDNA; the mixture incubated at 16°C for 1 h, and cDNA was purified using Ampure XP Beads (Beckman Coulter, Life Sciences, USA). The purified cDNA was supplemented with End-Repair Mix, incubated at 20°C for 30 min, and purified. The repaired cDNA was supplemented with A-Tailing mix and incubated at 37°C for 30 min. Then, ligation reaction was done by combining adenylated cDNA with adapters and ligation mix at 20°C for 20 min. Finally, PCR products were purified using Ampure XP Beads. The resulting cDNA library was quantified using an Agilent 2100 Bioanalyzer, Agilent DNA 1000 Reagent, and quantitative PCR (TaqMan Probe) (Fig 1).

**Fig 1:** cDNA library construction for transcriptome analysis of fat body tissues from *Rhynchophorus ferrugineus*.

### Transcriptome sequencing and *de novo* assembly

Competent libraries were amplified using cBot, and clusters generated on TruSeq PE Cluster Kit V3-cBot-HS; Illumina, a flow cell, were sequenced using Illumina HiSeq 2000 system. Read lengths were 50 bp and were sequenced via a paired-end strategy. The raw reads produced by the sequencing machine contained unclean reads (adapter contaminated, low quality, or containing unknown bases); the raw reads were cleaned using filter-fq to generate high-quality transcriptome data. The assembly was then created from the clean reads using assembling program Trinity (Version: release-20130225) [30]. Briefly, Trinity assembles clean reads into contigs, clusters the resulting contigs so that contigs of the same genes are grouped together, and then assembles the contigs into unigenes (Fig 2).

**Fig 2:** Diagram of the fat body tissues of *Rhynchophorus ferrugineus* unigene clusters assembly process.

### Unigene annotation

Assembled unigenes were aligned to different protein databases such as: non-redundant (NR), Swiss-Prot, Kyoto Encyclopedia of Genes and Genomes (KEGG), and Clusters of Orthologous Groups (COG) databases through the BLASTX tool (E-value < 0.00001) and to the nucleotide database (NT) using the BLASTN tool (E-value < 0.00001). The alignment results with the best sequence similarity were selected and annotated to the unigene. For unigenes that failed to align with the aforementioned databases, ESTScan software was used to detect the coding region sequence and to find the sequence direction [31]. Blast2GO software was used with NR annotation to obtain Gene Ontology (GO) term annotation (i.e., biological process, cellular component, and molecular function) [32]. After obtaining the GO annotation, GO functional classification was deduced for all unigenes using WEGO software [33]. To envisage and classify possible functions, unigenes were aligned with the COG database.

### SSR and SNP detection

All types of SSR sequences (mono to penta-nucleotide repeats) were identified using the software program MicroSAtellite (MISA), and only the SSRs in unigenes of >150 bp in length were retained. Similarly, all potential SNPs were identified and classified using the software program SOAPsnp [34].

### Identification of red palm weevil reproduction control genes

The genes involved in RPW reproduction were acknowledged from RPW fat body transcriptome data. The sequences of these genes were downloaded separately, and their identification was confirmed using the BLASTX tool from NCBI.

### Identification of the Vg genes and their validation through RT-PCR

Five Vg transcripts were identified from RPW transcriptome data with different FPKM values and validated via RT-PCR using following gene-specific primers: RfVgF1, RfVgR1, RfVg1F1, RfVg1R1, RfVg2F1, RfVg2R1, RfVg3F1, RfVg3R1, RfVg4F1, and RfVg4R1; actin primers RfActF1 and RfActR1 were used for normalization control (Table 1). Total RNA was extracted, cDNA library was synthesized and PCR was done by using the Gene Amp PCR system 9700 thermo-cyclers (Applied Biosystems, USA), under given conditions: (94°C, 1 min, followed by 35 cycles of 94°C, 30 s, and 68°C, 2 min). The PCR-amplified products were run on 1.5% agarose gel, stained with ethidium bromide, and visually confirmed using BioDocAnalyze, Biometra, gel documentation system.

**Table 1:** List of primers used for confirmation of the identified *RfVg* genes via RT-PCR.

Primers	Sequences
RfVgF1	5**′** TCTGGGGAGTAGCTCTAGCTTCGAT 3**′**
RfVgR1	5**′** CTGCCTACGTTTTGTTCAGAGATCC 3**′**
RfVg1F1	5**′** CCCAACAATACGCTGCTTCTTACAC 3**′**
RfVg1R1	5**′** TCCTCATCTGATCGGAGAATAGCTG 3**′**
RfVg2F1	5**′** GCTACCAGGTTCAGTCAGTGCAAGT 3**′**
RfVg2R1	5**′** GGTCGATTTTAGGACGGCAGATAAC 3**′**
RfVg3F1	5**′** ATTCCTAGGATGTCTGCTGGAGCTT 3**′**
RfVg3R1	5**′** TGAGATCTGAGCTTCCAGGTCAAGT 3**′**
RfVg4F1	5**′** CGACAAACTGACTGTTCTCACCAGA 3**′**
RfVg4R1	5**′** TCTGGTGAGAACAGTCAGTTTGTCG 3**′**
RfActF1	5**′** GACATCAGGGTGTCATGGTTGGTAT 3**′**
RfActR1	5**′** ATGGATACCACAAGCTTCCATACCC 3**′**

### Phylogenetic relationship of *RfVg* with other known insect Vgs

The sequence of *RfVg* was checked against the NCBI GenBank database using the BLASTX tool. The Vg amino acid sequences acquired from different insect species were used to construct a phylogenetic tree. Similarity analyses of the protein sequences were conducted. A multiple-sequence alignment was performed using the ClustalW program [35], and a neighbor-joining phylogenetic tree was constructed using MEGA 6.0 [36].

## Results

### Transcriptome sequencing and sequence assembly

In this study, 105,938,182 raw reads were generated from the RPW fat body cDNA library using the Illumina Hiseq 2000. After trimming adapter sequences and eliminating low-quality reads, the raw data yielded 102,645,544 clean reads and 9,238,098,960 clean nucleotides (nt), with a GC content of 40.31% (Table 2). From the processed data, 64,046 contigs were produced, with a total length of 30,808,342 nt and mean length of 481 nt. These contigs were set into 43,789 unigenes, with 51,342,530 nt and 1,172 nt bases for total length mean length, respectively (Figs 3 and 4).

**Fig 3:** Length distribution of contig sequences from the transcriptome data of *Rhynchophorus ferrugineus* fat body tissues. Nucleotide sequence size (nt) and number of contigs are shown on the X- and Y-axes, respectively.

**Fig 4:** Length distribution of unigene sequences from transcriptome data of *Rhynchophorus ferrugineus* fat body tissues. Nucleotide sequence size (nt) and number of unigenes are shown on the X- and Y-axes, respectively.

**Table 2:** Summary of the *Rhynchophorus ferrugineus* fat body tissue transcriptome.

Total raw reads	Total clean reads	Total clean nucleotides (nt)	Q20%	N %	GC %
105,938,182	102,645,544	9,238,098,960	98.68%	0.01%	40.31%

### Structural and functional annotation

The assembled unigene transcripts were annotated using public databases NR, Swiss-Prot, KEGG, and COG (E-value < 0.00001) with BLASTX, and the nucleotide database (NT; E-value < 0.00001) with BLASTN. Of the 43,789 unigenes, a total of 23,880 (54.53%) were annotated, including 23,178 (52.93%) using NR, 12,589 (28.74%) using NT, 18,706 (42.71%) using Swiss-Prot, 16,512 (37.7%) using KEGG, 9604 (21.93%) using COG, and 10,300 (23.52%) using GO databases (Table 3). Among 23,178 NR annotated unigenes, 3,739 were annotated exclusively with NR database, whereas the rest of the unigenes also shared annotation with other databases. Similarly, 21, 24, and 1 unigene were exclusively annotated with the Swiss-Prot, KEGG, and COG databases, respectively. Nearly 2,576 unigenes were annotated with NR and Swiss-Prot databases, whereas 709 were annotated with NR and KEGG databases. Furthermore, 6,553 were commonly annotated with NR, Swiss-Prot, and KEGG databases, and 354 were commonly annotated using the NR, Swiss-Prot, and COG databases. Additionally, 9,195 unigenes were annotated using all four protein databases (Fig 5).

**Fig 5:** Venn diagram of annotated unigenes from the *Rhynchophorus ferrugineus* fat body tissues transcriptome sequence using BLASTX (E-value < 0.00001) and protein databases Swiss-Prot, KEGG, NR, and COG.

**Table 3:** Summary of unigene annotation of the *Rhynchophorus ferrugineus* fat body tissues transcriptome.

Databases used for annotation	Number of unigenes	Annotated %
NR	23,178	52.93
NT	12,589	28.74
Swiss-Port	18,706	42.71
KEGG	16,512	37.7
COG	9,604	21.93
GO	10,300	23.52

In total, 23,178 unigenes shared resemblance to genes identified in the NR database. In the NR database sequence similarity of top hits with regard to E-value were, 67.3% sequences showing E-value of 0–60 and 20% of sequences with E-value of 80%–100% among sequences that possessed some homology (Fig 6A and 6B). The maximum proportion of homology sequences with other species in the NR database were from the mountain pine beetle *Dendroctonus ponderosae* (59.9%), followed by the red flour beetle *Tribolium castaneum* (26.9%) (Fig 6C).

**Fig 6:** E-value, sequence similarity, and species distribution of the *Rhynchophorus ferrugineus* fat body transcriptome sequences. (A) E-value distribution of top BLASTX hits against the non-redundant (NR) database for each unigene. (B) Sequence similarity distribution of the NR annotation results. (C) Species distribution of top BLASTX hits against the NR database.

The COG database classifies orthologous gene products, and each COG protein is presumed to come from an ancestral protein. In this study, unigenes were mapped to to predict possible functions using COG database. COG analysis permitted the functional classification of 9,604 unigenes (Fig 7).

**Fig 7:** Functional classification of unigenes from the *Rhynchophorus ferrugineus* fat body transcriptome according to COG criteria.

The most frequently identified class was “general function” (3,873), followed by “replication, recombination and repair” (1,840), “translation, ribosomal structure and biogenesis” (1,715), and “transcription” (1,439). In GO analysis, unigenes were separated into three ontologies: molecular function, cellular component, and biological process. GO analysis categorized 10,300 unigenes (23.52% of the total) into 60 functional groups. “Cellular process” and “metabolic process” were the 2 largest groups, containing 6,255 and 5,879 unigenes, respectively. However, “developmental process” and “reproduction” contained 1,540 and 536 unigenes, respectively (Fig 8).

**Fig 8:** Gene Ontology (GO) classification of identified unigenes from *Rhynchophorus ferrugineus* fat body tissues transcriptome. Functional classes “biological process,” “cellular components,” and “molecular function” are indicated by green, yellow, and red colors, respectively.

### Unigene KEGG pathway analysis

The unigene pathway analysis mapped 16,512 unigenes (37.7%) to 258 KEGG pathways. Metabolic pathways comprised 2,298 unigenes (13.91%), which was significantly more than the number mapped to other pathways, such as the pathways for the regulation of the actin cytoskeleton (615 unigenes, 3.72%), focal adhesion (532 unigenes, 3.22%), purine metabolism (508 unigenes, 3.08%), vascular smooth muscle contraction (473 unigenes, 2.86%), RNA transport (465 unigenes, 2.82%), cancer (464 unigenes, 2.81%), and the spliceosome (446 unigenes, 2.7%). According to KEGG classifications, there were six major annotational categories for the identified unigenes (Fig 9).

**Fig 9:** *Kyoto Encyclopedia of Genes and Genomes pathway annotation of the Rhynchophorus ferrugineus* fat body tissues transcriptome. Genes related to (A) metabolism, (B) cellular processes, (C) organismal systems, (D) genetic information processing, (E) diseases, and (F) environmental information processing were annotated.

### Protein coding region prediction

Unigenes were first aligned by BLASTX (E-value < 0.00001) to protein databases. The 22,861 coding DNA sequences (CDS) were mapped to protein databases, whereas, the EST scans predicted that 1,446 unigenes were related to CDS. However, 24,307 total numbers of CDS were obtained in the study (Figs 10 and 11).

**Fig 10:** Length distribution of unigenes from CDS of *Rhynchophorus ferrugineus* fat body tissues transcriptome data. Nucleotide sequence size (nt) and numbers of unigenes BLASTed are indicated on the X- and Y-axes, respectively.

**Fig 11:** Length distribution of EST scanned CDS from transcriptome data of *Rhynchophorus ferrugineus* fat body tissues. Nucleotide sequence size (nt) and numbers of unigene EST scans are indicated on the X- and Y-axes, respectively.

### SSR and SNP detection

Transcriptome analysis is an important source to develop genetic markers. In our study, a total of 2,060 SSRs were recognized (Table 4). The largest fraction of these was composed of dinucleotide repeat sequences (51.94%), followed by tri- (31.4%), mono- (14.51%), quad- (1.26%), and penta-nucleotide (0.82%) repeat sequences. Among the SSRs identified, the most abundant dinucleotide repeats were AT (40.09%) and TA (37.1%), accounting for 51.94% of the dinucleotide motifs, whereas the most abundant tri-nucleotide repeats were TTA (9.56%), ATC (6.63%), and ATA (5.24%), accounting for 31.4% of the tri-nucleotide motifs. Meanwhile, the most abundant repeat motifs were TTTA (26.92%) and TTTAT (23.52%).

**Table 4:** Summary of simple sequence repeats (SSRs).

SSR Type	No. of SSRs	Total SSRs (%)
Mono-nucleotides	299	14.51
Di-nucleotides	1,070	51.94
Tri-nucleotides	648	31.4
Quad-nucleotides	26	1.26
Penta-nucleotides	17	0.82
Hexa-nucleotides	0	0
Total	2060	100

In the transcriptome database, the present study identified a total of 59,012 high-quality SNPs, including 41,100 (69.64%) transitions and 17,912 (30.35%) transversions (Table 5). Together, A-to-G (34.61%) and C-to-T (35.03%) transitions were the most common SNPs and accounted for 69.64% of all SNPs identified. Among the transversions, A-to-T (9.33%) and A-to-C (7.16%) changes were the most common, followed by C-to-G (6.95%) and G-to-T (6.89%).

**Table 5:** Summary of SNPs (single nucleotide polymorphisms).

SNP Type	Count	Total (%)
Transition	41,100	69.64
A-G	20,428	34.61
C-T	20,672	35.03
Transversion	17,912	30.35
A-C	4,229	7.16
A-T	5,508	9.33
C-G	4,105	6.95
G-T	4,070	6.89
Total	59,012	100

### Red palm weevil reproduction control genes

The RPW reproduction control genes identified through the NCBI BLASTX tool are presented in Table 6. The putative identification showed that low density lipoprotein receptor gene consists of 6711 bp followed by Endoprotease Furin with 6578 bp. Moreover, there were several transcripts of *Vgs*, with maximum mean length of 5361 bp (unigene 12151). A variety of putative hormonal proteins that are involved in reproduction were also identified, including juvenile hormone-inducible protein, juvenile hormone epoxide hydrolase-like protein 5 precursor, juvenile hormone esterase, and ecdysone response nuclear receptor (Table 6).

**Table 6:** Reproduction control genes identified from the fat body tissues transcriptome of *Rhynchophorus ferrugineus*.

Unigene	Putative identification	Accession no.	Blast Hit score	**	*
				E-value	FPKM
Unigene12151	Vitellogenin	ALN38803	1839.3	0	5731.6087
Unigene11788	Vitellogenin	KY653077	123.6	5.00E-27	1.4716
Unigene19929	Vitellogenin	KY653076	114.8	2.00E-24	1.017
Unigene2157	Vitellogenin	KY307505	116.3	2.00E-21	1.028
Unigene11787	Vitellogenin	KY653078	159.1	1.00E-37	1.9639
Unigene21631	Apolipophorin III	KY407543	141	2.00E-30	0.7146
Unigene11367	Low-density lipoprotein receptor adapter protein 1	KY407544	232.3	8.00E-59	80.888
Unigene16398	Low-density lipoprotein receptor	KY407545	69.3	6.00E-09	83.2344
Unigene22552	minus strand s18 chorion protein	KY651032	58.5	2.00E-07	0.7189
Unigene16826	Endoprotease FURIN	KY407546	2123.6	0	6.9965
Unigene10592	Juvenile hormone-inducible protein	KY407547	340.5	2.00E-91	15.3077
Unigene13410	Juvenile hormone epoxide hydrolase-like protein 5 precursor	KY407548	563.1	2.00E-158	2298.6536
Unigene17335	Minus strand juvenile hormone esterase	KY407549	583.2	3.00E-164	24.0053
Unigene14301	Minus strand ecdysone receptor isoform A	KY407551	860.1	0	3.5593
Unigene14717	Similar to ecdysone response nuclear receptor	KY407551	1130.9	0	5.5027
Unigene9992	Similar to clathrin coat assembly protein	KY407552	377.9	8.00E-103	28.4123
Unigene6650	Minus strand NADH dehydrogenase flavoprotein 1	KY407553	182.6	9.00E-45	42.3405
Unigene17910	Dynein heavy chain	KY407554	577.8	4.00E-163	1.6786
Unigene21312	Prothoracicotropic hormone	KY653068	73.9	4.00E-12	0.8825
Unigene15690	Myosin-XVIIIa isoform 1	KY653069	2472.6	0	25.6146
Unigene10052	Mannose-P-dolichol utilization defect 1 protein homolog	KY653070	163.3	1.00E-38	49.3972
Unigene10459	Vesicular mannose-binding lectin	KY653071	366.3	1.00E-99	46.4972
Unigene10685	Transmembrane protein 59-like precursor	KY653073	247.7	1.00E-63	21.3118
Unigene12190	Proprotein convertase subtilisin/kexin type 4 furin	KY653074	1107	0	33.0508
Unigene16593	Macroglobulin complement-related CG7586-PA	KY653075	1212.6	0	8.8015

*Fragments per kilobase of transcript per million mapped reads.

**An expected value that reflect the sequence similarity.

### Identification of Vg genes and their validation through RT-PCR

The RPW fat body transcriptome data provided five partial *Vg* gene transcripts, one partial transcript was highly expressed with 5,731.60 FPKM value as compared with the other four (FPKM of 1.963, 1.471, 1.028, and 1.017, respectively), and were designated as *RfVg*, *RfVg1*, *RfVg2*, *RfVg3*, and *RfVg4*, respectively. The incongruity in the FPKM values of all five *Vg* transcripts was verified by RT-PCR, and expression was only confirmed of *RfVg* (Fig 12). A high expression level of *RfVg* was presumed on the basis of FPKM value, which was over 5,000 times that of the other 4 *Vg* genes, and RT-PCR analysis demonstrated that *RfVg* is the primary functional *Vg* gene in RPW.

**Fig 12:** The RT-PCR based confirmation of *RfVg* transcripts identified through transcriptome data. Agarose gel (2%) was used to analyze the amplified PCR products. M indicates the molecular-weight marker (bp). The size of the *RfVg* amplified products and actin genes are indicated on the right side.

### Phylogenetic relationship of *RfVg* with other insects

A neighbor-joining phylogenetic tree was constructed on the basis of known insect *Vg* sequences present in NCBI database to elucidate the evolutionary relationship of *RfVg* using the MEGA 6.0 program [36]. Phylogenetic analysis separated Coleopterans from species belonging to other groups and indicated that *RfVg* is more closely related to those of other Coleopterans, clustering with *Vg* of the boll weevil *Anthonomus grandis* (Fig 13). Phylogenetic analysis also suggested that sequence similarity is higher within this same group as compared with that in other groups.

**Fig 13:** Neighbor-joining phylogenetic tree of 80 insect Vgs representing 7 orders. The amino acid sequences were aligned using the ClustalW program and used as input for a neighbor-joining tree construction program (MEGA6) (Tamura et al. 2013). Scale 0.2 indicates distance (number of amino acid substitutions per site). Species belonging to different orders are indicated with bolls of different colors. *Gallus gallus* (representing galliformes) Vg was used as an out-group.

### Highly expressed genes in the red palm weevil fat body

The top 20 highly expressed transcripts in the RPW fat body based on FPKM value are summarized in Table 7. The most abundant transcripts included a hypothetical protein followed by ferritin, and transferrin. The *Vg*, a major yolk protein precursor, was also present among the highly expressed transcripts in RPW fat body tissues, thereby indicating its role in RPW reproduction.

**Table 7:** The highly expressed transcripts in *Rhynchophorus ferrugineus* fat body tissues transcriptome.

Unigene	Sequence description	E-value	FPKM
Unigene11341	Hypothetical protein	1.00E-08	78055.6231
Unigene11370	Hypothetical protein D910_04329	2.00E-51	49853.8746
Unigene4742	Hypothetical protein LOC100116930 isoform	6.00E-08	13247.3174
Unigene9720	Ferritin	1.00E-76	12884.1063
Unigene15223	Transferrin	0	9932.4045
CL428.Contig1	Elongation factor 1-alpha	0	9296.743
Unigene9707	Hypothetical protein YQE_03576, partial	1.00E-28	8870.8515
Unigene11369	Cytochrome c oxidase subunit III	1.00E-108	6580.6394
Unigene4741	Odorant-binding protein 28	4.00E-14	6531.4234
Unigene9536	Odorant-binding protein 9	2.00E-12	6401.9779
CL3374.Contig1	Cytochrome c oxidase subunit I	0	6315.9511
Unigene12151	Vitellogenin	0	5731.6087
Unigene9700	NADH dehydrogenase subunit 1	4.00E-113	4894.9444
Unigene12560	Cytochrome P450 CYP4g56	0	4806.6932
Unigene10790	Hypothetical protein YQE_05844, partial	2.00E-164	4605.3079
Unigene8942	Hypothetical protein YQE_03969, partial	2.00E-71	4141.3361
Unigene10950	Hypothetical protein YQE_11447, partial	3.00E-146	3668.2178
Unigene12206	Hypothetical protein YQE_08038, partial	5.00E-85	3271.7497
CL343.Contig4	Polyubiquitin-B	1.00E-36	3262.2426
Unigene4778	Odorant-binding protein 28	1.00E-22	3250.4219

*FPKM (fragments per kilobase of transcript per million mapped reads).

**E-value (an expected value that reflects the sequence similarity).

## Discussion

The RPW is the most critical pest of palm trees and causes severe damage as it spends its entire life cycle inside its host [37]. Despite an extensive range of control measures that have been applied to preclude and control RPW infestation [13–15, 38], none have proved to be successful, as the concealed nature of RPW reproduction within the palm trunk complicates efficient management. In addition, most of the research on RPW has focused on the species’ basic ecology and biology [10–12]. Thus, because of limited knowledge regarding molecular mechanisms of RPW reproduction is a major obstacle to further understand this species. Accordingly, the genes involved in the specie’s biological, physiological, and metabolic processes are primary goals for developing safer control strategies to combat this crucial pest of palm trees. The fat body plays a very critical role in metabolism, and one of its prominent roles is the storage and utilization of energy [39]. The transcriptome analysis represents RNA transcripts expressed in particular cells or tissues of an organism, and characterization of the identified transcripts is crucial to understand genome functional complexity, as well as the organism’s cellular activities related to reproduction, growth, and the immune response. Previously, the Illumina platform was only utilized for organisms with available reference genomes [16, 40–41]. However, recent technological advances have introduced the capability of *de novo* sequencing and the assembly of short genes into unigenes [42].

The Illumina sequencing of the RPW fat body yielded 102,645,544 clean reads, comprising 64,046 contigs and 43,789 unigenes (Table 2). Almost 54.53% (23,880) of the unigenes were significantly homologous with sequences in publicly available protein databases and are consistent with results reported previously [19, 43]. In addition, transcriptome data produced a greater number and lengths of unigenes than earlier transcriptome studies [21]. The mean unigene length and GC content were also similar to prior data [43], but the GC content was higher than that reported previously [21]. The present results indicated that RPW shares approximately 83.9% homology with other Coleopteran species, such as *Dendroctonus ponderosae* (56.7%) [28] and the red flour beetle *Tribolium castaneum* (27.2%).

In this research, most of the unigenes were annotated with COG and GO databases (9,604 and 10,300, respectively). The general function prediction class (3,873 unigenes, 40.32%) was the largest COG class, showing similarity to other insects transcriptome data [19, 43]. Among the GO categories (Fig 8), cellular process (2,255) and metabolic process (5,879) were the most abundant terms among biological processes, cell (3,916) and cell part (3,915) were the most abundant terms among cellular components, and catalytic activity (5,201) and binding (5,108) were the most abundant terms among molecular functions, as previously reported in case of insect transcriptome data [21, 43, 44]. In KEGG analysis, 16,512 unigenes mapped to 258 KEGG pathways, including metabolic pathways, the regulation of the actin cytoskeleton, focal adhesion, and purine metabolism (Fig 9). Among these, metabolic pathways were the most abundant (2,298 unigenes, 13.91%), as previously reported [19].

From the RPW fat body transcriptome, nearly 25 annotated genes were predicted to be involved in reproduction. Among these, *Vg* is one of the major gene which is highly expressed in RPW female fat bodies during reproductive phase and retain a substantial role in in oviparous organism’s reproduction [9, 29, 45–51]. The reproductive success of oviparous species depends on *Vg* production and accumulation in oocytes by membrane-bound receptors (the VgRs) via receptor-mediated endocytosis [8, 52–55]. Egg production is also increased with the increase in Vg production [56]. The accumulated egg yolk provides a nutritional reserve for the developing embryos, including proteins, carbohydrates, lipids, and phosphates [57–59]. In oviparous species, the yolk protein is mainly composed of vitellin (Vn). In the American cockroach *Periplaneta americana* [5, 60], German cockroach *Blattella germanica* [61], and yellow fever mosquito *Aedes aegypti* [62], Vn contributes approximately 88%, 93%, and 75%, of the total yolk protein, respectively.

In general, the *de novo* transcriptome sequence data in the present study demonstrate substantial homology to sequences in publicly available NCBI databases. This indicates that the Illumina-based transcriptome data of the present study were correctly assembled and that a significant fraction of exclusive genes was transcribed in RPW fat body tissues. From the present transcriptome data, five partial *Vg* gene transcripts were obtained; however, based on the FPKM values and RT-PCR results, it is very clear that *RfVg* is the only functional *Vg* gene in RPW. This is also in accordance with other Coleopteran species such as the boll weevil *Anthonomus grandis* [63], mealworm beetle *Tenebrio molitor* [64], nipa palm hispid beetle *Octodonta nipae* [65], and cabbage beetle *Colaphellus bowringi* [66], where a single *Vg* gene has been reported. Presence of different numbers of *Vg* genes in insect species have been recorded from several insect including *A*. *aegypti* [67, 68], the brown-winged green bug *Plautia stali* [69], *P*. *americana* [45, 46], and the Madeira cockroach *Leucophae maderae* [29, 70], only a single *Vg* gene has been depicted so far by members of the order Coleoptera [50]. Thus, our present findings, along with previous published information, conclusively demonstrate that RPW harbor only a single functional *Vg* gene. This current transcriptome data from RPW fat body tissues have delivered a surplus strong evidences regarding the genes involved in RPW physiological functions, especially in the reproduction. Reproduction control genes identification will make available a reference line for characterization of these genes. In particular, *Vg* gene characterization would be of great worth to understand RPW reproduction mechanism at molecular level and may encourage the biotech-based control strategies development against this pest species.

## Supporting information

S1 File (DOCX)
